# Combining Ability Analysis of Relevant Characters of Maize Inbred Lines Suitable for Machine Harvest

**DOI:** 10.1155/2022/2480801

**Published:** 2022-03-24

**Authors:** Long Jiang, Meiqi Rong, Mingxin Wang, Dianyuan Chen, Haiyan Yu

**Affiliations:** College of Agronomy, Jilin Agricultural Science and Technology University, Jilin 132101, Jilin Province, China

## Abstract

In this study, 9 maize inbred lines and 36 combinations were used as materials to analyze the combining ability of plant height, ear height, kernel depth, grain water content, tassel branches, stem diameter, and 100 kernels weight so as to screen excellent inbred lines and maize combinations with suitable mechanical harvest characters, which would provide a theoretical basis for breeding new maize varieties suitable for mechanical harvest. The results showed that JK2023, JK2368, and JK2018 were inbred lines whose comprehensive characters met the machine harvest standard and performed well. Besides, the combinations that meet the machine harvest standard and perform well were JK2023 × JK2197, JK2023 × JK2368, JK2023 × JK2005, JK2197 × JK2005, JK2197 × JK2368, and JK2368 × JK2005.

## 1. Introduction

Maize (*Zea mays* L.) is one of the important gramineous crops in China [1–3]. It is an important “ballast” to ensure national food security [1, 4]. It plays an important role in ensuring national food security and promoting industrial development [5, 6]. At present, the research and production technology of maize grain harvest in the United States and other countries was very mature, and the whole process mechanization has been realized [7, 8]. However, China started relatively late. Not only was the research on maize mechanized harvest not deep enough, the technology was not mature enough, but also the level of maize mechanization was very low [9]. Firstly, the lack of germplasm resources means there are few maize varieties suitable for mechanized harvest in the market [7]. Secondly, the research on the characteristics of maize suitable for mechanized harvesting was not deep enough [10]. Last but not least, the corn harvester and production technology were not mature enough [4, 11]. In recent years, scholars at home and abroad have done some research on the characteristics of suitable harvest characters of maize [11–14]. We should start with the selection of maize plants with lodging resistance and other aspects [15]. In addition to the uniformity and lodging resistance of maize plants, plant height and ear height were also important traits that affected the adaptability of maize to mechanical harvest [16]. Plant height was of great significance to the economic yield of maize [17]. The stem thickness, plant height, and ear height of maize would all affect the lodging resistance of the plant, and the stem thickness was the key factor [10]. The number of branches in the male ear was less, which was also an important condition to meet the mechanization of maize [16]. Maize grain water content was also an important index affecting machine harvest [18]. The dehydration rate of maize was controlled by a variety of agronomic characters, such as plant stem diameter, plant height, ear height, 100 kernel weights, and so on [19]. The results of previous studies showed that the main factors affecting the mechanized harvest of maize were the lodging resistance of the maize plant and the grain water content at harvest. Plant height, ear height, and stem diameter were the key factors affecting lodging, and kernel depth and 100 kernel weights were the main factors affecting grain water content. Therefore, this experiment analyzed the variance of the combining ability of plant height, ear height, and machine harvest characters of maize inbred lines and combinations and estimated the genetic parameters of each character. Thus, excellent inbred lines and combinations suitable for cultivating mechanized harvesting maize were selected, which provided a reference for breeding new varieties of maize suitable for mechanized harvesting.

## 2. Materials and Methods

### 2.1. Plant Materials

The maize inbred lines in this study were provided by the maize genetic breeding team of Jilin Agricultural Science and Technology University. The names and characteristics of inbred lines were shown in Table 1. In 2020, 36 combinations were prepared from 9 inbred lines according to NC II genetic design.

### 2.2. Experimental Design

In 2021, inbred lines and combinations were planted in the maize breeding experimental site of Jilin Agricultural Science and Technology University. This experiment adopted a randomized block design, with a total of 3 repetitions and 4 rows. The length of each district was 4 m, and the row spacing was 0.65 m. Field management was the same as other maize fields.

During the maize filling period, 10 representative plants were selected from each experimental plot, and then their plant height, ear height, plant stem diameter, and the number of branches of male ears were measured and recorded. The water content was measured after harvesting maize ears in the autumn. After drying, 10 maize ears were selected for an indoor seed test. The ear diameter and shaft diameter of the ears were measured, and the maize grain depth was calculated.

### 2.3. Data Analysis

SPSS was used to analyze the variance of maize kernel character data. And the program of Griffing combining ability analysis, method IV, was used to analyze the variance of combining ability and estimate the genetic parameters of each trait [8].

## 3. Results and Analysis

### 3.1. Variance Analysis of Relevant Characters Suitable for Machine Harvest

The variance analysis of six characters, including stem diameter, ear height, plant height, and so on, is shown in Table 2. The results showed that the plant stem diameter, ear height, and water content at harvest of the six suitable mechanical harvest characters among different combinations reached significant levels. Therefore, it is known that a genetic difference exists in the tested combinations, and the combining ability variance of 6 characters needs to be further analyzed.

### 3.2. Variance Analysis of Combining Ability of Suitable Harvest Correlation

The combining ability of 6 characters of the tested combinations was analyzed by variance (Table 3). The results showed that there were significant differences in the six suitable mechanical harvest characters of the tested combinations. Therefore, it was necessary to analyze the variance of general combining ability effect and special combining ability effect of six traits.

### 3.3. GCA Effect Analysis of Suitable Harvest Traits

General combining ability effect analysis *F* values of 9 tested materials are shown in Table 4. The results showed that the general combining ability effect value of plant stem diameter of inbred lines JK2018, JK2023 and JK2368 showed an obvious positive effect, which was conducive to promoting stem thickening and was suitable for breeding varieties with high lodging resistance. The plant height and ear height of inbred lines JK2018, JK2023, and JK2368 showed obvious negative effects, which were conducive to the combination of varieties with lower plant height and ear height. The tassel branch number of inbred lines JK2023, JK2130, JK2197, and JK2368 showed an obvious negative effect, which was conducive to breeding varieties with fewer tassel branches. The inbred lines JK2018, JK2023, JK2368, and JK2005 showed a significant positive effect on grain depth, which made them suitable to be used as parents of combinations with kernel depth. The grain water content at harvest of inbred lines JK2018, JK2023, and JK2368 showed a significant negative effect, indicating that these three inbred lines were conducive to reducing the grain water content of hybrid combinations. Considering the general combining ability effect values of six traits, JK2018, JK2023, and JK2368 were the most suitable inbred lines as parents among the tested inbred lines.

### 3.4. SCA Effect Analysis of Suitable Harvest Traits

The special combining ability effect values of 36 tested combinations were listed in Table 5. The results showed that the combinations JK2001 × JK2368, JK2001 × JK2368, JK2018 × JK2130, JK2023 × JK2197, JK2023 × JK2368, JK2023 × JK2005, JK2197 × JK2368, JK2197 × JK2005, JK2198 × JK2005, and JK2368 × JK2005 had a significant positive effect on the relative effect value of the special combining ability of stem diameter, which was suitable for the combination of relative lodging resistance. The relative effect values of the special combining ability of plant height and ear height of combinations JK2001 × JK2368, JK2023 × JK2197, JK2023 × JK2368, JK2023 × JK2005, JK2197 × JK2368, JK2197 × JK2005, and JK2368 × JK2005 showed obvious negative effects, which were conducive to reducing the plant height and ear height of maize hybrids. Special combining ability, relative effect value of the number of male panicle branches of the hybrid combinations JK2018 × JK2005, JK2368 × JK2005, JK2023 × JK2368, JK2197 × JK2368, JK2023 × JK2197, JK2198 × JK2368, JK2023 × JK2005, and JK2197 × JK2005 showed a significant negative effect. It was easier to use them to prepare a combination with relatively few tassel branches. The relative effect value of the special combining ability of water content at harvest of combinations JK2023 × JK2197, JK2018 × JK2023, JK2197 × JK2368, JK2001 × JK2198, JK2197 × JK2005, JK2197 × JK2411, JK2023 × JK2368, and JK2368 × JK2005 showed a significant negative effect, which showed that they were more suitable for combining maize varieties with low water content.

The yield results of 36 combinations are shown in Table 6. The results showed that the yield of combinations JK2197 × JK2368, JK2023 × JK2197, JK2197 × JK2005, JK2023 × JK2005, JK2368 × JK2005, JK2023 × JK2368, JK2001 × JK2005, and JK2130 × JK2005 were in the top eight. The comprehensive analysis of the effect value of the special combining ability of six characters showed that six combinations, including JK2023 × JK2197, JK2023 × JK2368, JK2023 × JK2005, JK2197 × JK2368, JK2197 × JK2005, and JK2368 × JK2005 were more in line with the machine harvest standard.

### 3.5. Genetic Parameter Analysis of Relevant Traits Suitable for Machine Harvest

The estimated values of the genetic parameters of each trait are shown in Table 7. The results showed that the variance of general combining ability and special combining ability of stem diameter accounted for 50% of the variance, which showed that stem diameter was controlled by additive and nonadditive genes. The variance of general combining ability of plant height, ear height, tassel branch, and water content at harvest was much greater than that of special combining ability, indicating that these traits are inherited through additive effect genes. The variance of general combining ability at grain depth is much smaller than that of special combining ability, indicating that kernel depth is greatly affected by nonadditive genetic effects. The estimated value of genetic parameters of environmental variance of plant height and ear height was large, indicating that plant height and ear height were easily affected by environmental factors. Because the broad-sense heritability and narrow-sense heritability of tassel branch and water content at harvest are relatively high, and the additive effect of a gene was greater than that of a nonadditive effect, it was less affected by environmental factors, so it was suitable to select in the early generation. Plant height and ear height were easily affected by environmental factors, so they were suitable for selection in the late generation. The broad-sense heritability and narrow-sense heritability of kernel depth are higher, and they are greatly affected by nonadditive effects, so they can be selected in the late generation.

## 4. Conclusion and Discussion

The development of maize mechanization is conducive to promoting the development of China's agriculture, and one of the conditions restricting the development of mechanization is that there are few varieties of maize suitable for machine harvest [4, 20]. At present, the breeding methods of maize varieties suitable for machine harvest in China mainly focus on improving maize plant agronomic characters [12]. Previous experiments showed that the combination of parents with high general combining ability may not have high special combining ability, while the combination of parents with low general combining ability or one high and one low may also obtain high special combining ability [21]. This view was consistent with the results of this experiment. Therefore, if we want to breed a variety combination suitable for mechanized harvest of maize, we need to fully understand the parental characters first [22]. Then, extensive test crossing experiments on parents can be carried out to select maize combinations suitable for mechanized harvest of maize.

In this experiment, the inbred lines JK2018, JK2023, and JK2368 had high general combining ability and conformed to the characteristics suitable for machine harvest. They were the preferred inbred lines of machine harvested maize and were suitable to be used as the parents of varieties with lodging resistance and low water content. JK2023 × JK2197, JK2023 × JK2368, JK2023 × JK2005, JK2197 × JK2368, JK2197 × JK2005, and JK2368 × JK2005 had high special combining ability and relatively meets the standard of mechanical harvest. It was necessary to further determine and analyze the characteristics of grain filling rate, dehydration rate, and bract characters of these six maize combinations [23]. On this basis, the adaptability of varieties was identified so as to better screen out maize suitable for mechanical harvest [24, 25]. Based on the above analysis, it could be concluded that the inbred lines meeting the machine harvest standard were JK2023, JK2368, and JK2018. The combinations that meet the machine harvest standard were JK2023 × JK2197, JK2023 × JK2368, JK2023 × JK2005, JK2197 × JK2005, JK2197 × JK2368, and JK2368 × JK2005 [26].

## Figures and Tables

**Table 1:** Characteristics of 9 inbred lines.

Inbred lines	Consanguinity	Plant shape	Plant height	Ear height	Stem diameter	Water content at harvesting	Tassel branch	100 kernel weight
JK2001	*Lan*	Loose	272.1	161	1.9	27	4	36.9
JK2005	*Reid*	Compact	257.3	107	2.7	24	8	43.6
JK2018	*Reid*	Compact	245.4	108	2.6	20	6	39.7
JK2023	*Lan*	Compact	241.2	105	2.7	21	8	40.3
JK2130	*Reid*	Loose	172.9	96	1.8	29	11	29.8
JK2197	*Reid*	Compact	250.8	111	2.6	24	6	41.8
JK2198	*Reid*	Loose	210.7	100	2.0	26	10	31.6
JK2368	*Lan*	Compact	246.9	102	2.8	20	6	43.9
JK2411	*Reid*	Loose	290.5	186	1.9	29	8	36.5

**Table 2:** Analysis of variance of 6 characters of 36 combinations (*F* value).

Variance source	DF	Plant shape	Plant height (cm)	Stem diameter (cm)	Tassel branch (cm)	Kernel depth (cm)	Water content at harvesting (%)
Between groups	2	13.52	30.00	0.05	0.58	5.25	2.32
Between combinations	35	13.97^*∗∗*^	3.65^*∗*^	1.61^*∗*^	27.56^*∗∗*^	11.64^*∗∗*^	95.04^*∗∗*^

Note: ^*∗*^indicated a significant difference (*P* < 0.05), ^*∗∗*^indicated an extremely significant difference (*P* < 0.01). It indicates the same in the tables that follow.

**Table 3:** Variance analysis of combining ability of 6 characters of 36 combinations (*F* value).

Source of variation	DF	Plant height (cm)	Ear height (cm)	Stem diameter (cm)	Tassel branch (cm)	Kernel depth (cm)	Water content at harvesting (%)
GCA	8	44.18^*∗∗*^	11.46^*∗∗*^	4.41^*∗∗*^	91.51^*∗∗*^	16.50^*∗∗*^	287.35^*∗∗*^
SCA	27	5.03^*∗∗*^	0.15^*∗∗*^	0.81^*∗∗*^	8.62^*∗∗*^	10.20^*∗∗*^	38.06^*∗∗*^

**Table 4:** GCA effect values of 6 characters of 9 inbred lines.

Inbred lines	Plant height (cm)	Ear height (cm)	Stem diameter (cm)	Tassel branch (cm)	Kernel depth (cm)	Water content at harvesting (%)
JK2001	12.4221^*∗∗*^	8.7216^*∗∗*^	0.0016	0.2592	0.1685	−0.1893
JK2005	−17.7967^*∗∗*^	11.4544^*∗∗*^	0.0049	1.8306^*∗∗*^	0.4208^*∗*^	1.2655^*∗∗*^
JK2018	−12.0491^*∗∗*^	−4.2877^*∗*^	0.0685^*∗∗*^	2.2645^*∗∗*^	0.5091^*∗∗*^	−1.1369^*∗∗*^
JK2023	−14.9110^*∗∗*^	−4.9782^*∗*^	0.0690^*∗∗*^	−0.7121^*∗*^	0.3756^*∗*^	−0.5131^*∗∗*^
JK2130	5.4269	3.6978^*∗*^	−0.0227	−1.8835^*∗∗*^	−0.8054^*∗∗*^	1.3057^*∗∗*^
JK2197	29.0983^*∗∗*^	8.2551^*∗∗*^	−0.0152	−0.8361^*∗*^	−0.0743	1.4821^*∗∗*^
JK2098	−1.5586	2.0925	−0.1289^*∗∗*^	2.1163^*∗∗*^	−1.0885^*∗∗*^	0.2676^*∗*^
JK2368	−12.9872^*∗∗*^	−5.6211^*∗∗*^	0.0723^*∗∗*^	−1.1692^*∗∗*^	0.8327^*∗∗*^	−0.8703^*∗∗*^
JK2411	9.3555^*∗*^	2.5597	−0.0298	2.2592^*∗∗*^	−0.1385	0.2400^*∗∗*^
LSD_0.05_	8.6585	2.6603	0.0421	0.6731	0.3468	0.2387
LSD_0.01_	11.4984	5.0079	0.0620	0.8937	0.4607	0.3162

**Table 5:** SCA effect values of 6 characters of 36 combinations.

Combinations	Plant height (cm)	Ear height (cm)	Stem diameter (cm)	Tassel branch (cm)	Kernel depth (cm)	Water content at harvesting (%)
JK2001 × JK2018	−1.5225	0.4059	−0.0479	0.5001	0.6536	1.3416^*∗∗*^
JK2001 × JK2023	2.8678	1.6059	0.0781	1.7380^*∗*^	−0.3142	0.9511^*∗∗*^
JK2001 × JK2130	12.3392	2.4963	0.0234	−0.4523	0.3666	−0.2297
JK2001 × JK2197	−7.1178	−5.1844	−0.0012	0.8332	0.3928	1.5606^*∗∗*^
JK2001 × JK2198	3.3201	3.1059	−0.0755	0.9761	0.6499	−0.7725^*∗∗*^
JK2001 × JK2368	−17.5893^*∗*^	−5.6344^*∗∗*^	0.0972^*∗*^	0.5475	−0.2713	1.0773^*∗∗*^
JK2001 × JK2411	7.2535	5.7820^*∗*^	−0.1184^*∗*^	0.1666	0.3404	0.9368^*∗∗*^
JK2001 × JK2005	11.3441	5.7061^*∗*^	−0.0407	0.5951	−1.8001^*∗∗*^	−0.2963
JK2018 × JK2023	−0.4511	4.8963	0.0143	0.5951	−0.2309	−0.9201^*∗∗*^
JK2018 × JK2130	9.2535	2.1535	0.0895^*∗*^	0.0713	−1.2001^*∗∗*^	−0.4011
JK2018 × JK2197	−5.9701	2.0059	−0.0384	2.6427^*∗∗*^	0.4760	0.4561
JK2018 × JK2198	4.4725	1.3441	−0.0041	1.6904^*∗*^	−0.0108	0.4559
JK2018 × JK2368	7.7154	4.6963	0.0614	0.0712	−0.9380^*∗∗*^	0.5177^*∗*^
JK2018 × JK2411	−13.3987	−4.6941	−0.0355	−1.0752	−0.5761	0.0986
JK2018 × JK2005	14.3582	−1.4035	0.0221	−1.4523^*∗*^	−0.5501	0.5486^*∗*^
JK2023 × JK2130	5.1441	−0.0130	0.0024	−0.0237	−0.7501^*∗*^	2.1416^*∗∗*^
JK2023 × JK2197	−20.5752^*∗*^	−11.4463^*∗∗*^	0.0895^*∗*^	−1.7380^*∗*^	1.1404^*∗∗*^	−0.5013^*∗*^
JK2023 × JK2198	−7.7703	−0.3894	−0.0512	1.7380^*∗*^	0.6668	−0.2010
JK2023 × JK2368	−17.4082^*∗*^	−5.4273^*∗*^	0.0905^*∗*^	−1.8332^*∗∗*^	0.5715^*∗*^	−1.4868^*∗∗*^
JK2023 × JK2411	4.4820	7.4752^*∗*^	−0.0403	0.5002	−0.0261	1.2416^*∗∗*^
JK2023 × JK2005	−18.7415^*∗*^	−5.7082^*∗*^	0.1002^*∗*^	−1.3494^*∗*^	0.7666^*∗*^	1.6820^*∗∗*^
JK2130 × JK2197	4.3582	8.7297^*∗*^	−0.0036	0.7380	−0.0427	0.8178^*∗∗*^
JK2130 × JK2198	3	0.9676	−0.0026	0.0713	−5.0356^*∗∗*^	−0.3154
JK2130 × JK2368	1.2201	2.3822	−0.0117	−0.5475	−1.2094^*∗*^	−0.1201
JK2130 × JK2411	−5.2368	−3.0035	0.0157	0.9761	0.2047	1.6701^*∗∗*^
JK2130 × JK2005	−18.7130^*∗*^	13.7130^*∗∗*^	−0.1130^*∗*^	−0.8332	−1.3474^*∗∗*^	0.2130
JK2197 × JK2198	9.9773	4.5868	−0.0664	2.0237^*∗∗*^	−1.1570^*∗∗*^	1.2751^*∗∗*^
JK2197 × JK2368	−18.9701^*∗*^	−5.3654^*∗*^	0.0924^*∗*^	−1.7380^*∗*^	0.7475^*∗*^	−0.8062^*∗∗*^
JK2197 × JK2411	−6.5942	−4.7511	−0.0055	0.4047	−0.2198	−0.5392^*∗*^
JK2197 × JK2005	−19.9963^*∗*^	−5.4273^*∗*^	0.1285^*∗*^	−1.4142^*∗*^	0.8761^*∗*^	−1.7105^*∗∗*^
JK2198 × JK2368	18.0059^*∗*^	4.8058	0.1310^*∗∗*^	−1.5951^*∗*^	−0.7594^*∗*^	−0.2344
JK2198 × JK2411	−4.5176	3.8535	0.0744	2.5950^*∗∗*^	−1.2715^*∗∗*^	1.2169^*∗∗*^
JK2198 × JK2005	8.7725	−3.7225	0.1200^*∗*^	0.4523	0.5477	1.4367^*∗∗*^
JK2368 × JK2411	26.4335^*∗∗*^	3.4011	−0.0072	−0.0236	−0.5511	1.9222^*∗∗*^
JK2368 × JK2005	−37.8415^*∗∗*^	−6.0248^*∗*^	0.1026^*∗*^	−1.9284^*∗∗*^	0.8094^*∗*^	−1.1963^*∗∗*^
JK2411 × JK2005	11.3678	5.8392^*∗*^	0.0642	0.6903	−0.4454	1.4796^*∗∗*^
LSD_0.05_	17.3176	5.3210	0.0844	1.3468	0.6946	0.4764
LSD_0.01_	22.9976	10.0180	0.1203	1.7878	0.9214	0.6328

**Table 6:** The yield of 36 combinations.

Combinations	kg/667 m^2^	Combinations	kg/667 m^2^	Combination	kg/667 m^2^
JK2001 × JK2018	499.24	JK2018 × JK2368	485.56	JK2130 × JK2411	587.45
JK2001 × JK2023	532.12	JK2018 × JK2411	472.59	JK2130 × JK2005	595.65
JK2001 × JK2130	541.38	JK2018 × JK2005	579.54	JK2197 × JK2198	546.39
JK2001 × JK2197	483.36	JK2023 × JK2130	581.49	JK2197 × JK2368	660.10
JK2001 × JK2198	469.76	JK2023 × JK2197	647.72	JK2197 × JK2411	559.68
JK2001 × JK2368	476.87	JK2023 × JK2198	577.35	JK2197 × JK2005	626.66
JK2001 × JK2411	5702.85	JK2023 × JK2368	608.24	JK2198 × JK2368	492.24
JK2001 × JK2005	596.84	JK2023 × JK2411	590.85	JK2198 × JK2411	481.64
JK2018 × JK2023	588.51	JK2023 × JK2005	622.22	JK2198 × JK2005	571.12
JK2018 × JK2130	481.68	JK2130 × JK2197	581.84	JK2368 × JK2411	597.56
JK2018 × JK2197	521.25	JK2130 × JK2198	575.25	JK2368 × JK2005	605.52
JK2018 × JK2198	577.52	JK2130 × JK2368	578.25	JK2411 × JK2005	584.87

**Table 7:** Estimated values of genetic parameters of various traits.

Genetic parameters	Plant height (cm)	Ear height (cm)	Stem diameter (cm)	Tassel branch (cm)	Kernel depth (cm)	Water content at harvesting (%)
Environmental variance (%)	113.13	77.34	0.03	0.67	0.47	0.17
GCA variance (%)	73.48	84.39	50.00	75.64	16.32	65.78
SCA variance (%)	26.52	15.61	50.00	24.36	83.68	34.22
Generalized heritability (%)	83.53	51.90	25.75	91.26	78.58	97.30
Narrow heritability (%)	61.38	46.35	25.75	69.03	12.83	63.97

## Data Availability

The datasets used in this paper are available from the corresponding author upon request.

## References

[1] Han Y. (2022). Theoretical logic, historical logic and practical logic of China’s food security strategy. *Reforma*.

[2] Yu H. Y., Li K. H. (2021). Global food security governance and China’s participation. *The Journal of International Studies*.

[3] Sun J.-Y., Gao J.-L., Yu X.-F. (2018). Combining ability of sixteen USA maize inbred lines and their outbreeding prospects in China. *Agronomy*.

[4] Qiu H. G., Li X. H., Yu J. L. (2021). China maize industry: development trends and policy suggestions. *Issues in Agricultural Economy*.

[5] Wang K. R., Xie R. Z., Ming B., Hou P., Xue J., Li S. K. (2021). Review of combine harvester losses for maize and influencing factors. *International Journal of Agricultural and Biological Engineering*.

[6] Wang Y., Gao L. L. L. S., Li L. (2020). Evaluation of grain breakage sensitivity of maize varieties mechanically-harvested by combine harvester. *International Journal of Agricultural and Biological Engineering*.

[7] Wang Z. H., Lu X. M., Zhang X., Zhang Q. J., Wei X. (2011). Analysis of maize breeding objective from full mechanization in China. *Journal of Henan Agricultural Sciences*.

[8] Yu Y. X., Liu J. L., Jia L. (2018). Combining ability of maize inbred lines for traits related to appropriate mechanical harvesting. *Journal of Maize Sciences*.

[9] Wang C. Y., Shu Z. Z., Cheng B. J., Jiang H. Y., Li X. Y. (2018). Advances and perspectives in maize mechanized harvesting in China. *Journal of Anhui Agricultural University*.

[10] Yan S. F., Liu H. F., Sun S. K. (2017). The effects of correlative factors on stem lodging resistance in maize. *Molecular Plant Breeding*.

[11] Guo Y. Q., Xu W. J., Wang K. R. (2021). Actuality and factors influencing farmer adoption of mechanized harvesting in typical maize ecoregions. *Chinese Journal of Eco-Agriculture*.

[12] Yu R. S., Tian X. K., Liu B. B. (2022). Dissecting the genetic architecture of lodging related traits by genome-wide association study and linkage analysis in maize. *Acta Agronomica Sinica*.

[13] Li S. K., Wang K. R., Chu Z. D. (2019). Study on the current status of maize mechanical kernel harvest and the hultivar characteristics in the 1-3 accumulated temperature zones in Heilongjiang province. *Journal of Maize Sciences*.

[14] Wang R., Xu T., Zhao J. (2020). Effects of harvest date on maize grain moisture content and grain mechanical harvesting quality. *Journal of Agricultural Science and Technology*.

[15] Chen D. Y., Jing X. Q., Wang X. J., Cao Z. B. (2014). Discussion on the breeding for mechanical harvesting and density tolerant maize hybrids. *Crops*.

[16] Tang W. M., Zhao C. H., Yang H., Tong S. H. (2015). Requirement and strategy for breeding in maize production mechanization. *Horticulture&Seed*.

[17] Tollenaar M., Lee E. (2002). Yield potential, yield stability and stress tolerance in maize. *Field Crops Research*.

[18] Chai Z. W., Wang K. R., Guo Y. Q. (2017). Current status of maize mechanical grain harvesting and its relationship with grain moisture content. *Scientia Agricultura Sinica*.

[19] Xie L. H., Gao H., Zhang X. Y., Chen M. L., Liu M. (2020). Study on the main agronomic characters affecting dehydration of maize varieties for machine harvesting in Heilongjiang province. *Heilongjiang Agricultural Sciences*.

[20] Li S., Wang K., Xie R. (2016). Implementing higher population and full mechanization technologies to achieve high yield and high efficiency in maize production. *Crops*.

[21] Li H. T., Wang J., Zhang S. H., Chi M., Wang D. M., Hu J. (2015). Heterosis and combining ability of plant height and its components of barley. *Acta Agriculturae Zhejiangensis*.

[22] Zhu Y. G., Han T., Dou D. D., Wang H. T., Ku L. X., Chen Y. H. (2017). Combining ability analysis on dehydration rate in later stage of maize harvest mechanization. *Journal of Maize Sciences*.

[23] Cui T., Fan C. L., Zhang D. X., Yang L., Li Y. B., Zhao H. H. (2019). Research progress of maize mechanized harvesting technology. *Transactions of the Chinese Society for Agricultural Machinery*.

[24] Cao Y. J., Sha S., He W. J. (2020). Influence factors of machine harvest maize grains and the cultivation regulation: research progress. *Chinese Agricultural Science Bulletin*.

[25] Yan S. Q., Su J., Li C. X. (2007). Combining ability of grain filling rate in maize. *Journal of Maize Sciences*.

[26] Zhengwan Z., Chunjiong Z., Hongbing L. I., Tao X. (2020). Multipath transmission selection algorithm based on immune connectivity model. *Journal of Computer Applications*.

